The article "MicroRNA-122-3p plays as the target of long non-coding RNA LINC00665 in repressing the progress of arthritis" was retracted in 2026. Reasons: concerns about the data; concerns about the results or conclusions.

# MicroRNA-122-3p plays as the target of long non-coding RNA LINC00665 in repressing the progress of arthritis

**DOI:** 10.1080/21655979.2022.2081757

**Published:** 2022-05-29

**Authors:** Zhiyan Wang, Qijun Tian, Yumei Tian, Zhonghua Zheng

**Affiliations:** a Department of Rheumatology, Shouguang People’s Hospital, Shouguang, Shandong, P.R. China; b Trauma orthopedics, The No. 4 hospital of Jinan, Jinan, Shandong, P.R. China; c School of Nursing, Hunan University of Medicine, Huaihua, Hunan, P.R. China; d Department of Teaching Supervision and Evaluation, JILin Medical University, Jilin, Jilin, P.R. China

**Keywords:** Rheumatoid arthritis, miR-122-3p, LINC00665, EIF2AK1, mTOR signaling pathway

## Abstract

MicroRNAs (miRNAs) play important roles in many diseases, including rheumatoid arthritis (RA). However, the mechanisms underlying the effects of miR-122-3p-3p on RA are not distinct and require further investigation. Patients with RA and healthy controls were recruited to analyze the miR-122-3p levels. The MH7A cells were stimulated with interleukin (IL)-1β to mimic the local inflammation of RA. Cell Counting Kit-8 (CCK-8) and flow cytometry were performed to measure the viability and apoptosis of MH7A cells. Diana tools and TargetScan were used to predict the target relationships. Luciferase reporter assay was used to validate the target relationship. miR-122-3p is downregulated in RA patients and IL-1β-stimulated MH7A cells. miR-122-3p suppresses MH7A cell viability and promotes MH7A cell apoptosis. miR-122-3p targets LINC00665. LINC00665 eliminates the inhibitory effect of miR-122-3p on IL-1β-stimulated MH7A cells. Eukaryotic translation initiation factor 2 alpha kinase 1 (EIF2AK1) targets miR-122-3p. In addition, EIF2AK1 is highly expressed in patients with RA. In addition, EIF2AK1 activates the mTOR signaling pathway. miR-122-3p represses RA progression by reducing cell viability and increasing synoviocyte apoptosis.

## Highlights

- miR-122-3p reduced cell viability of IL-1β-induced MH7A cells
- miR-122-3p is a target gene of LINC00665
- miR-122-3p directly target to EIF2AK1
- LINC00665 regulates EIF2AK1 expression by targeting miR-122-3p
- LINC00665 activates the mTOR pathway by regulating EIF2AK1 in MH7A cells

## Introduction

Rheumatoid arthritis (RA), characterized by symmetrical peripheral polyarthritis, can result in joint destruction and may be related to extra-articular features [1,2]. It affects approximately 1% of the global population [3]. It also burdens patients concerning their life and occupations due to bone and cartilage damage and an unsatisfactory rate of full remission [4,5]. RA is genetically susceptible, and the risk of developing RA in patients with a family history is higher, and the heritability of seropositive RA is as high as 40%-65% [4]. Several studies have shown that miRNAs play considerable roles in RA pathogenesis [2,6,7].

The article "MicroRNA-122-3p plays as the target of long non-coding RNA LINC00665 in repressing the progress of arthritis" was retracted in 2026. Reasons: concerns about the data; concerns about the results or conclusions.

Many microRNAs (miRNAs) are tissue-specific and are related to various diseases, such as arthritis [8]. Bi X et al. found that miR-4701-5p inhibited the proliferation of fibroblast-like synoviocytes (FLSs) in RA [9]. miR-17-5p plays an anti-inflammatory and anti-erosive role in RA [10]. In addition, Wang et al. found that miR-122-3p was expressed at low levels in the plasma of patients with RA [11]. miR-122 is involved in the proliferation and apoptosis of synoviocytes in osteoarthritis [12]. However, the mechanism of action of miR-122-3p in RA has not yet been elucidated.

Long noncoding RNAs (lncRNAs) have been reported to play crucial roles in RA [13,14]. LOC100506036 is involved in RA inflammation by regulating SMPD1 and NFAT1 [15]. LncRNA PICSAR knockdown significantly inhibited proliferation of RA-FLSs cells [9]. Studies have demonstrated that LINC00665 is involved in the progression of breast cancer, lung adenocarcinoma, and osteosarcoma [16–19]. It is worth noting that LINC00665 was highly expressed in spinal cord injury (SCI) rats and LPS-induced PC12 cells [20]. Therefore, it is worth studying whether LINC00665 affects RA progression.

This study aimed to investigate the role of miR-122-3p in RA and further reveal the underlying mechanisms in RA. In this study, miR-122-3p was expressed at low levels in RA synovial tissues and IL-1β-stimulated FLSs. miR-122-3p inhibited cell viability and facilitated apoptosis of IL-1β-stimulated MH7A cells.

## Materials and methods

### Specimens

A total of 16 RA and nine non-RA fresh synovial tissues and peripheral blood samples were obtained from our hospital. Gene expression was measured by qRT-PCR. The protocol has been approved by the Ethics Committee of Shouguang People’s Hospital (20,201,103). All patients have signed written informed consent.

### Bioinformatic analysis

The target relationship between LINC00665 and miR-122-3p was analyzed using the Diana tools software. The interaction between miR-122-3p and EIF2AK1 was analyzed using TargetScan. GSEA was used to analyze the impact of EIF2AK1 on signaling pathways based on the GEO dataset GSE94519 [21].

### IL-1β treatment

MH7A cells were purchased from EK-Bioscience (Shanghai, China). MH7A cells were cultured in DMEM added with 10% FBS at 37°C with 5% CO_2_. Different concentrations of IL-1β (1, 5, and 10 ng/ml) were used to stimulate MH7A cells for 24 h to simulate local inflammation in RA [22].

### Transfection

The miR-122-3p mimic, inhibitor, and NC were purchased from GenePharma (Shanghai, China). MH7A cells were transfected with miR-122-3p mimic/inhibitor and NC using Lipofectamine 2000 (Carlsbad, CA, USA) [23].

The article "MicroRNA-122-3p plays as the target of long non-coding RNA LINC00665 in repressing the progress of arthritis" was retracted in 2026. Reasons: concerns about the data; concerns about the results or conclusions.

### qRT-PCR

Total RNA was extracted from the cells using TRIzol reagent (Shanghai Generay Biotech Co., Ltd). Reverse transcription of total RNA was performed using a PrimeScript® RT Reagent Kit (TaKaRa, Beijing, China). The SYBR Green PCR Mastermix (Carlsbad, CA, USA) was used for qPCR. U6 and GAPDH served as the internal controls for LINC00665, miR-122-3p, and EIF2AK1, respectively. The relative expression levels of LINC00665, miR-122-3p, and EIF2AK1 were calculated using the 2-ΔΔCt method. Primer sequences were synthesized by Sangon Biotech (Shanghai, China) as follows: LINC00665 (5’-AGCACCCCTAGTGTCAGT CA-3’, forward; 5’-TGGTCTCTAGGGAGGCAGAA-3’, reverse); has-miR-122-3p (5’-AGCACCCCTAGTGTCAGT CA-3’, forward; 5’-TGGTCTCTAGGGAGGCAGAA-3’, reverse); EIF2AK1 (5’-TCAGTTTGCCTTCCTGGATTT-3’, forward; 5’-TCTTCCCGTATCCTGGTTGG-3’, reverse); GAPDH (5’-CATGAGAAGTATGACAACAGCCT-3’, forward; 5’-AGTCCTTCCACGATACCAAAGT-3’, reverse); U6 (5’-CTCGCTTCGGCAGCACA-3’, forward; 5’-AACGCTTCACGAATTTGCGT-3’, reverse) [24].

### Western blotting

Total protein was isolated by RIPA lysis buffer (Thermo Fisher Scientific). Protein samples were separated by 10% SDS-PAGE and transferred to a PVDF membrane. Thereafter, the membranes were incubated with primary antibodies at 4°C overnight. Blots were detected using an ECL kit (Thermo Fisher Scientific) [25].

### CCK-8 assay

The cells were cultured in 96-well plates (1× 10^3^ cells/well). After 48 h of culture, CCK-8 reagent was added into the 96-well plates and incubated 2 h at 37°C. Absorbance was measured at 450 nm using a microplate reader [26].

### Cell apoptosis

Cells at a density of 1 × 10^6^/ml were mixed with Annexin V/FITC (5 μl) and PI (5 μl). After incubation in the dark at room temperature for 15 min, the FlowJo software was used to analyze the apoptotic rates of the cells [27].

### Dual luciferase reporter assay

The 3’-UTR sequences, including LINC00665-WT or LINC00665-Mut (or EIF2AK1-WT and EIF2AK1-Mut) were cloned into the PGL3 reporter plasmid. LINC00665 (or EIF2AK1) plasmids were co-transfected with miR-122-3p mimic or mimic NC into cells. Luciferase activity was detected using a dual-luciferase reporter assay system [28].

### RNA pull‑down assay

miR-122-3p, miR-122-3p-mutant (miR-122-3p Mut) with disrupted base pairing between LINC00665 and miR-122-3p or its negative control (NC) were purchased from GenePharma (Shanghai, China). miRNAs were biotin-labeled using the Biotin RNA Labeling Mix (Roche, Basel, Switzerland) and T7/SP6 RNA polymerase (Roche). Whole cell lysates were mixed and incubated with biotinylated RNAs. The complexes were then incubated with Streptavidin agarose beads (Invitrogen) for 1 h at 37°C. The beads were washed, and RNA level were analyzed by qRT-PCR [29].

The article "MicroRNA-122-3p plays as the target of long non-coding RNA LINC00665 in repressing the progress of arthritis" was retracted in 2026. Reasons: concerns about the data; concerns about the results or conclusions.

### Statistical analysis

Data were analyzed using GraphPad Prism and expressed as the mean ± SD. Differences were analyzed using Student’s t-test or one-way ANOVA followed by Tukey’s post hoc test. P < 0.01 was considered as significant difference.

## Results

This study was conducted to establish RA cell models in MH7A cells using IL-1β treatment and transfection of miR-122-3p mimic or inhibitor into MH7A cells. Subsequent findings revealed that miR-122-3p was expressed at low levels in IL-1β-treated MH7A cells, whereas the miR-122-3p mimic increased IL-1β-induced apoptosis inhibition. In addition, we explored the mechanism of miR-122-3p and found that miR-122-3p was a target of LINC00665 and inhibited EIF2AK1, thus removing IL-1β-induced apoptosis inhibition to alleviate RA.

### The effects of miR-122-3p in IL-1β-stimulated MH7A cells

miR-122-3p levels were lower in RA synovial tissues and peripheral blood than those in normal tissues and peripheral blood (Figure 1a). In addition, the viability of MH7A cells increased after exposure to different concentrations of IL-1β (5 ng/ml and 10 ng/ml) (Figure 1b). The miR-122-3p level was decreased by IL-1β treatment (Figure 1c). Thus, IL-1β at 10 ng/ml was used to stimulate MH7A cells to establish an RA model in vitro in the following studies.

**Figure 1.** **miR-122-3p inhibited apoptosis of IL-1β-treated MH7A cell**. (a) The qRT-PCR for the expression of miR-122-3p in synovial tissues and peripheral blood samples of patients without RA or with RA. (b) CCK-8 assay for the cell viability of M7HA cells stimulated with different concentrations of IL-1β (1 ng/ml, 5 ng/ml, and 10 ng/ml). (c) QRT-PCR for the expression of miR-122-3p in MH7A cells stimulated with different concentrations of IL-1β (1 ng/ml, 5 ng/ml, and 10 ng/ml). (d) The qRT-PCR for the miR-122-3p level in M7HA cells. **P < 0.01. (e) CCK-8 assay for the cell viability of MH7A cells. (f) Flow cytometric analysis for apoptosis. (g) Western blotting for the levels of Bax, Bcl-2, and cleaved caspase-3. **P < 0.01 vs. control group, ##P < 0.01 vs. IL-1β+mimic NC group. (h) The qRT-PCR for the miR-122-3p expression in M7HA cells. **P < 0.01. (i) CCK-8 assay for the cell viability of MH7A cells. (j) Flow cytometric analysis for apoptosis of MH7A cells. (k) Western blotting for the levels of Bax, Bcl-2, and cleaved caspase-3 in MH7A cells. **P < 0.01 vs. control group, ##P < 0.01 vs. IL-1β+inhibitor NC group.

The article "MicroRNA-122-3p plays as the target of long non-coding RNA LINC00665 in repressing the progress of arthritis" was retracted in 2026. Reasons: concerns about the data; concerns about the results or conclusions.

To further verify the potential influence of miR-122-3p in RA, the miR-122-3p mimic and its NC were transfected into cells. The miR-122-3p level was significantly increased in miR-122-3p mimic-transfected cells (Figure 1d), indicating successful transfection of MH7A cells. Thereafter, we examined the cell viability and apoptosis. Cell viability was markedly reduced in the IL-1β+miR-122-3p mimic group than in the IL-1β+mimic NC group (Figure 1e). Cell apoptosis is significantly reduced by IL-1β treatment. miR-122-3p significantly facilitated apoptosis in IL-1β-treated MH7A cells (figure 1f). In addition, as shown in Figure 1g, IL-1β treatment significantly enhanced Bcl-2 levels and reduced the levels of Bax and cleaved caspase-3. The miR-122-3p mimic significantly inhibited Bcl-2 expression while promoting the expression of Bax and cleaved caspase-3 in IL-1β-induced cells (Figure 1g). Furthermore, the miR-122-3p levels were significantly decreased by miR-122-3p inhibitor (Figure 1h). The miR-122-3p inhibitor markedly increased cell viability (Figure 1i) and decreased apoptosis (Figure 1j) in IL-1β-stimulated cells. Compared to the IL-1β+inhibitor NC group, the miR-122-3p inhibitor significantly increased Bcl-2 levels and decreased the levels of Bax and cleaved caspase-3 (Figure 1k).

### miR-122-3p is a target of lncRNA LINC00665 in MH7A cells

The target genes of miR-122-3p in RA were analyzed using Diana tools software. The results showed binding sites between miR-122-3p and LINC00665 (Figure 2a). The target relationship between them was verified by dual-luciferase reporter and RNA pull-down assays (Figure 2 b and c). qRT-PCR analysis suggested that LINC00665 was highly expressed in RA patients (Figure 2d). In addition, IL-1β treatment significantly increased LINC00665 expression (Figure 2e). LINC00665 expression was enhanced by LINC00665 overexpression and decreased by LINC00665 siRNAs treatment (figure 2f). We measured miR-122-3p expression after LINC00665 overexpression and silencing. miR-122-3p level was markedly reduced by LINC00665 overexpression and increased by LINC00665 silencing (Figure 2g).

**Figure 2.** **miR-122-3p was a target of LINC00665 in MH7A cells**. (a) The Diana tools were used for the binding sites between LINC00665 and miR-122-3p. (b) Luciferase reporter activity. (B) RNA pull-down assay to confirm the target relationship between LINC00665 and miR-122-3p. (d) The qRT-PCR to detect LINC00665 level in tissues. (e) QRT-PCR to detect LINC00665 in IL-1β (10 ng/ml) treated MH7A cells. (f) QRT-PCR to detect LINC00665 level in MH7A cells. (g) QRT-PCR to detect miR-122-3p expression in MH7A cells after transfection with LINC00665 overexpressed plasmid and LINC00665 siRNAs. **P < 0.01.

The article "MicroRNA-122-3p plays as the target of long non-coding RNA LINC00665 in repressing the progress of arthritis" was retracted in 2026. Reasons: concerns about the data; concerns about the results or conclusions.

### LINC00665 eliminates the inhibited effect of miR-122-3p on MH7A cells

Thereafter, miR-122-3p mimic (or inhibitor) and LINC00665 pcDNA3.1 (or siRNA) were co-transfected to evaluate the effect of LINC00665 on MH7A cells. LINC00665 overexpression increased cell viability and eliminated the influence of miR-122-3p mimic on cell viability (Figure 3a). As shown in Figure 3b, LINC00665 overexpression significantly decreased apoptosis and eliminated the effect of the miR-122-3p mimic on MH7A cell apoptosis. In addition, LINC00665 overexpression increased Bcl-2 levels but decreased Bax and cleaved caspase-3 levels (Figure 3c). Furthermore, LINC00665 silencing significantly inhibited cell viability, accelerated apoptosis, inhibited Bcl-2 levels, increased the levels of Bax and cleaved caspase-3, and eliminated the effect of miR-122-3p inhibitor on MH7A cells (Figure 3d**~F**).

**Figure 3.** **LINC00665 eliminates the inhibited effect of miR-122-3p on MH7A cells**. (a) CCK-8 assay to detect cell viability of MH7A cells after transfection with miR-122-3p mimic and LINC00665 overexpressed plasmid. (b) Flow cytometric analysis for apoptosis of IL-1β treated MH7A cells. (c) Western blotting for Bax, Bcl-2, and cleaved caspase-3 expression in MH7A cells. **P < 0.01 vs. Vector group, ##P < 0.01 vs. mimic NC group, &&P < 0.01 vs. miR-122-3p group. (d) CCK-8 assay for cell viability of MH7A cells after co-transfection with miR-122-3p inhibitor and LINC00665 siRNA. (e) Flow cytometric analysis for apoptosis of IL-1β treated MH7A cells. (f) Western blotting for the levels of Bax, Bcl-2, and cleaved caspase-3 in IL-1β treated MH7A cells. **P < 0.01 vs. si-NC group, ##P < 0.01 vs. inhibitor NC group, &&P < 0.01 vs. miR-122-3p inhibitor group.

### MiR-122-3p directly targets 3′UTR of EIF2AK1 in MH7A cells

Further analysis based on TargetScan showed that EIF2AK1 was a target gene of miR-122-3p (Figure 4a), and the dual luciferase reporter assay confirmed the target relationship between them (Figure 4b). EIF2AK1 was upregulated in RA synovial tissues and IL-1β stimulated M7HA cells (p < 0.001, Figure 4 c and d). Furthermore, we found that EIF2AK1 levels were markedly decreased by the miR-122-3p mimic and significantly increased by the miR-122-3p inhibitor (Figure 4 e and f).

**Figure 4.** **EIF2AK1 is a target gene of miR-122-3p**. (a) TargetScan was used for miR-122-3p target gene analysis. (b) Luciferase reporter activity in MH7A cells. **P < 0.01 vs. mimic NC group. (C/D) The EIF2AK1 expression in RA tissues and cells. (E/F) The EIF2AK1 expression in MH7A cells. **P < 0.01.

### LINC00665 regulates EIF2AK1 expression by targeting miR-122-3p

We analyzed the correlation between LINC00665, miR-122-3p, and EIF2AK1 expression using Spearman’s correlation method. miR-122-3p expression was negatively correlated with LINC00665 and EIF2AK1 levels in RA synovial tissues (Figure 5a, b). LINC00665 expression positively correlated with EIF2AK1 expression (Figure 5c). In addition, we found that the expression of EIF2AK1 was markedly increased by LINC00665 overexpression (Figure 5d). The miR-122-3p mimic significantly reduced the effect of LINC00665 overexpression on EIF2AK1 expression (Figure 5d). LINC00665 silencing significantly decreased EIF2AK1 expression, and this inhibitory effect was eliminated by the miR-122-3p inhibitor (Figure 5e).

The article "MicroRNA-122-3p plays as the target of long non-coding RNA LINC00665 in repressing the progress of arthritis" was retracted in 2026. Reasons: concerns about the data; concerns about the results or conclusions.

**Figure 5.** **LINC00665 regulates EIF2AK1 expression by targeting miR-122-3p**. (a) The correlationship between LINC00665 and miR-122-3p. (b) The correlationship between LINC00665 and EIF2AK1. (c) The correlationship between miR-122-3p and EIF2AK1. (D/E) The EIF2AK1 expression in MH7A cells. **P < 0.01 vs. Vector group, ##P < 0.01 vs. pc-LINC00665+ mimic NC group.

### LINC00665 silence eliminates the promoted effect of EIF2AK1 overexpression on MH7A cells

EIF2AK1 pcDNA3.1 (or siRNA) and LINC00665 siRNA (or pcDNA3.1) were co-transfected to evaluate the effect of EIF2AK1 on MH7A cells. ELF2AK1 expression was significantly increased by EIF2AK1 overexpression (Figure 6a). Compared to the Vector group, EIF2AK1 overexpression increased cell viability and decreased cell apoptosis (Figure 6 b and c). As shown in Figure 6d, EIF2AK1 overexpression significantly increased Bcl-2 levels but decreased Bax and cleaved caspase-3 levels. However, the effects of EIF2AK1 overexpression on MH7A cells were eliminated by the LINC00665 siRNA. The effects of EIF2AK1 siRNA on MH7A cells were also investigated. EIF2AK1 levels were significantly decreased by EIF2AK1 siRNAs treatment (Figure 6e). EIF2AK1 silencing remarkably inhibited cell viability, accelerated apoptosis, inhibited Bcl-2 levels, and increased Bax and cleaved caspase-3 levels (figure 6f, H). LINC00665 overexpression eliminated the effect of EIF2AK1 silencing in MH7A cells (figure 6f, H).

**Figure 6.** **LINC00665 silence eliminates the promoted effect of EIF2AK1 overexpression on MH7A cells**. (a) QRT-PCR and western blotting were used to measure EIF2AK1 expression in MH7A cells after transfection with EIF2AK1 overexpressed plasmid. (b) CCK-8 assay to detect cell viability of MH7A cells after transfection with EIF2AK1 overexpressed plasmid and LINC00665 siRNA. (c) Flow cytometric analysis for apoptosis of IL-1β treated MH7A cells. (d) Western blotting for Bax, Bcl-2, and cleaved caspase-3 expression in MH7A cells. **P < 0.01 vs. Vector group, ##P < 0.01 vs. pc-EIF2AK1+ si-NC group. (e) QRT-PCR and western blotting were used to measure EIF2AK1 expression in MH7A cells after transfection with EIF2AK1 siRNAs (f) CCK-8 assay for cell viability of MH7A cells after co-transfection with EIF2AK1 siRNA and LINC00665 overexpressed plasmid. (g) Flow cytometric analysis for apoptosis of IL-1β treated MH7A cells. (h) Western blotting for the levels of Bax, Bcl-2, and cleaved caspase-3 in IL-1β treated MH7A cells. **P < 0.01 vs. si-NC group, ##P < 0.01 vs. si-EIF2AK1#1+ Vector group.

The article "MicroRNA-122-3p plays as the target of long non-coding RNA LINC00665 in repressing the progress of arthritis" was retracted in 2026. Reasons: concerns about the data; concerns about the results or conclusions.

### LINC00665 activates the mTOR pathway by regulating EIF2AK1 in MH7A cells

To identify the mechanism of EIF2AK1 in RA, we performed GSEA using GEO dataset GSE94519. The results revealed that EIF2AK1 activated the mTOR signaling pathway (Figure 7a). Thereafter, we measured the protein expression of the mTOR pathway after EIF2AK1 overexpression or silencing. EIF2AK1 significantly increased the levels of p-mTOR/mTOR and PGF, whereas the opposite results were obtained in EIF2AK1-silenced cells (Figure 7 b and c). Figure 7d shows that LINC00665 overexpression markedly increased the levels of p-mTOR/mTOR and PGF. The levels of p-mTOR/mTOR and PGF were markedly decreased in the pc-LINC00665+ miR-122-3p mimic group compared to those in the pc-LINC00665+ mimic NC group. In addition, the inhibitory effect of miR-122-3p on the mTOR pathway was eliminated by EIF2AK1 overexpression. LINC00665 silencing significantly reduced the levels of p-mTOR/mTOR and PGF (Figure 7e). The miR-122-3p inhibitor eliminated the inhibitory effect of LINC00665 silencing on the mTOR pathway. Compared to the si-LINC00665+ miR-122-3p inhibitor group, the levels of p-mTOR/mTOR and PGF in the si-LINC00665+ miR-122-3p inhibitor+si-EIF2AK1 group were significantly decreased (P < 0.01).

**Figure 7.** **LINC00665 activates the mTOR pathway by regulating EIF2AK1 in MH7A cells**. (a) The analysis of Gene set enrichment analysis (GSEA) showed that EIF2AK1 activated mTOR signaling pathway. (b) Western blotting for the levels of p-mTOR/mTOR and PGF in MH7A cells after transfection with EIF2AK1 overexpressed plasmid. **P < 0.01 vs. Vector group. (c) Western blotting for the levels of p-mTOR/mTOR and PGF in MH7A cells after transfection with EIF2AK1 siRNA. **P < 0.01 vs. si-NC group. (d) Western blotting for the levels of p-mTOR/mTOR and PGF in MH7A cells after co-transfection with LINC00665 overexpressed plasmid, miR-122-3p mimic, and EIF2AK1 overexpressed plasmid. **P < 0.01 vs. Vector group, ##P < 0.01 vs. pc-LINC00665+ mimic NC group, &&P < 0.01 vs. pc-LINC00665+ miR-122-3p mimic group. (e) Western blotting for the levels of p-mTOR/mTOR and PGF in MH7A cells after transfection with LINC00665 siRNA, miR-122-3p inhibitor, and EIF2AK1 siRNA. **P < 0.01 vs. si-NC group, ##P < 0.01 vs. si-LINC00665+ inhibitor NC group, &&P < 0.01 vs. si-LINC00665+ miR-122-3p inhibitor group.

The article "MicroRNA-122-3p plays as the target of long non-coding RNA LINC00665 in repressing the progress of arthritis" was retracted in 2026. Reasons: concerns about the data; concerns about the results or conclusions.

## Discussion

Rheumatoid arthritis invades the synovium of the affected joint, causes synovitis and pannus formation, and triggers articular cartilage damage, eventually leading to cartilage and bone destruction and disability [30]. Therefore, it is necessary to investigate the role of miR-122-3p in the pathogenesis of RA and explore efficient treatment methods for RA.

In this study, miR-122-3p expression was significantly decreased in RA synovial tissues. IL-1β is an important mediator of inflammatory responses and is upregulated in autoimmune diseases including RA [31]. We treated MH7A cells with IL-1β to mimic the local inflammation of RA. miR-122-3p expression was decreased by IL-1β. The miR-122-3p mimic inhibited cell viability and accelerated apoptosis of RA cells. In contrast, the miR-122-3p inhibitor has the opposite effect. It has been reported that miR-122 exhibits anti-inflammatory effects in the liver [32]. The miR-122 mimic reduces the cell proliferation of osteoarthritis synoviocytes [12]. The results of our study were consistent with those of previous studies. These findings showed that miR-122-3p might inhibit RA progression by suppressing cell viability and promoting synoviocyte apoptosis.

Growing evidence suggests that lncRNAs contribute to RA [33]. LncRNA PlncRNA-1 overexpression mediates the upregulation of TGF-β1 in RA synovial fibroblasts [34]. Studies have indicated that lncRNAs can competitively bind to miRNAs and act as ceRNAs [35]. Silencing of lncRNA PICSAR inhibited the viability of RA FLSs by targeting miR-4701-5p [9]. LncRNA MEG3 was downregulated in RA FLSs compared with healthy subjects, and the inhibitory effects of lncRNA MEG3 were partially abolished by overexpression of miR-141 [36]. This study found that LINC00665 acts as a ceRNA in RA. LINC00665 was highly expressed in RA synovial tissues and cells. LINC00665 overexpression enhanced cell viability and reduced apoptosis of RA cells, whereas LINC00665 silencing markedly reduced cell viability and accelerated apoptosis. In addition, the effects of LINC00665 overexpression on RA FLSs were eliminated by miR-122-3p overexpression. Similarly, the inhibitory effects of LINC00665 silencing were eliminated by the miR-122-3p inhibitor. These data show that the protective effect of miR-122-3p on RA might be regulated by LINC00665.

Eukaryotic translation initiation factor 2 alpha kinase 1 (EIF2AK1) is a member of the EIF2AK family [37]. EIF2AK1 corresponds to haeme deprivation and proteasome inhibition to maintain basal stress in endoplasmic reticulum [38–40]. Moreover, EIF2AK1 contains two heme-binding sites and two protein kinase domains [37]. EIF2AK1 was identified as a target gene of some miRNAs (such as miR-129, −145, −155), which have been shown to function in glioma cell growth [41]. We found that EIF2AK1 is a target gene of miR-122-3p and that it is highly expressed in RA synovial tissues. In addition, IL-1β treatment increased EIF2AK1 expression. EIF2AK1 levels were negatively correlated with miR-122-3p and positively correlated with LINC00665 expression. The expression of EIF2AK1 was enhanced by LINC00665 overexpression and reduced by the miR-122-3p mimic. The above data showed that EIF2AK1 may be participate in RA progression as a target of miR-122-3p.

The article "MicroRNA-122-3p plays as the target of long non-coding RNA LINC00665 in repressing the progress of arthritis" was retracted in 2026. Reasons: concerns about the data; concerns about the results or conclusions.

The mTOR signaling pathway is involved in RA [42,43]. Du et al. showed that mTOR pathway is activated in TNF-α-treated RA FLSs [44]. Rapamycin, an mTOR inhibitor, efficiently alleviates synovial hyperplasia in rats with RA [45]. MEG3 plays a protective role in RA by deactivating the mTOR signaling pathway [36]. In this study, EIF2AK1 was found to activate the mTOR signaling pathway. EIF2AK1 overexpression significantly increased the levels of p-mTOR/mTOR and PGF levels. In addition, we found that the expression of p-mTOR/mTOR and PGF was increased by LINC00665 overexpression and decreased by miR-122-3p mimic. Thus, we speculated that the protective effect of miR-122-3p on RA might be achieved through the mTOR pathway regulated by EIF2AK1.

## Conclusion

In summary, our findings indicated that miR-122-3p effectively ameliorates RA progression via sponging LINC00665. Moreover, miR-122-3p regulates the mTOR signaling pathway by inhibiting EIF2AK1 expression. A limitation of this study is the lack of further studies on the role of EIF2AK1 in regulating the mTOR pathway in RA.

## Supplementary Material

Supplemental Material

## Data Availability

The datasets used and/or analysed during the current study are available from the corresponding author on reasonable request.
